The article "Optimal Deep Learning-Based Vocal Fold Disorder Detection and Classification Model on High-Speed Video Endoscopy" was published in 2022. Journal: J Healthc Eng.

# Optimal Deep Learning-Based Vocal Fold Disorder Detection and Classification Model on High-Speed Video Endoscopy

**DOI:** 10.1155/2022/4248938

**Published:** 2022-10-17

**Authors:** S. Sakthivel, V. Prabhu

**Affiliations:** ^1^Department of Computer Science and Engineering, Vel Tech High Tech Dr. Rangarajan Dr. Sakunthala Engineering College, Avadi, Chennai, India; ^2^Department of Electronics and Communication Engineering, Vel Tech Multi Tech Dr. Rangarajan Dr. Sakunthala Engineering College, Chennai, India

## Abstract

The use of high-speed video-endoscopy (HSV) in the study of phonatory processes linked to speech needs the precise identification of vocal fold boundaries at the time of vibration. The HSV is a unique laryngeal imaging technology that captures intracycle vocal fold vibrations at a higher frame rate without the need for auditory inputs. The HSV is also effective in identifying the vibrational characteristics of the vocal folds with an increased temporal resolution during retained phonation and flowing speech. Clinically significant vocal fold vibratory characteristics in running speech can be retrieved by creating automated algorithms for extracting HSV-based vocal fold vibration data. The best deep learning-based diagnosis and categorization of vocal fold abnormalities is due to the usage of HSV (ODL-VFDDC). The suggested ODL-VFDDC technique starts with temporal segmentation and motion correction to identify vocalized regions from the HSV recording and gathers the position of movable vocal folds across frames. The attributes gathered are fed into the deep belief network (DBN) model. Furthermore, the agricultural fertility algorithm (AFA) is used to optimize the hyperparameter tuning of the DBN model, which improves classification results. In terms of vocal fold disorder classification, the testing results demonstrated that the ODL-VFDDC technique beats the other existing methodologies. The farmland fertility algorithm (FFA) is then used to accurately determine the glottal limits of vibrating vocal folds. The suggested method has successfully tracked the speech fold boundaries across frames with minimum processing cost and high resilience to picture noise. This method gives a way to look at how the vocal folds move during a connected speech that is completely done by itself.

## 1. Introduction

In recent years, higher-speed video endoscopy (HSV) has been used to objectively analyze the vibratory properties of the vocal folds during both continuous phonation and flowing speech [1]. Unlike the visual stroboscope, HSV is a powerful tool for understanding the complicated physiological and phonological factors that govern sound output. HSV records vocal cord movements and has become a prominent method for detecting voice issues [1]. An examination of the vocal cords is a part of the medical evaluation of the voice. However, in medical situations, acoustic analysis has remained the most useful tool for studying glottal aerodynamics and providing information on speaker voice function. The acoustic parameter is devoid of bias and gives a quantitative evaluation of perceived voice quality [2]. In order to gather meaningful data on the supra-glottal glottis and glottal source, visual data of the vocal fold must be included. HSV offers some benefits over alternative approaches. The vocal waveform may be collected and analyzed to get high-quality data on vocal fold motion and glottal airflow variations over time [3].

The article "Optimal Deep Learning-Based Vocal Fold Disorder Detection and Classification Model on High-Speed Video Endoscopy" was published in 2022. Journal: J Healthc Eng.

HSV is especially beneficial for quantifying and visualizing disorders that influence the dynamics of vocal folds [4]. Voice computation is a valuable technique for evaluating intracycle and cycle-to-cycle vibratory properties, as well as nonstationary phonation activities [5]. However, without the assistance of computerized research tools, sifting through the huge amount of data acquired by employing HSV is impossible in medical practice. Because of advancements in automated algorithms for extracting HSV-enabled measurements of vocal fold vibration [6], users may now get medically appropriate vocal fold vibratory features while running speech. Machine learning (ML) methods are required for mining large HSV data sets. Using this ML method and at a lower processing cost, we could classify and identify hidden patterns or similar and dissimilar structures in the data more efficiently. Several of the methods used in the study could also be used to find and categorize diseases [7].

The disease diagnosis in this method is based on an automatic categorization judgment, but there is no apparent sign of the presence of a voice problem. An automated system user could diagnose the sickness more accurately and precisely if supported by visual signs. The bulk of today's advanced devices is designed to detect vocal fold problems [8]. Some approaches rely on calculating F0, which is a difficult issue in and of itself due to the nonperiodic nature of disordered speech signals [9]. Each artificial neural network (ANN) contains a vast number of layers that aid in the processing of data, and each hidden layer may have a particular activation function. The hidden layer tries to reach more goals, but it is not the product's final “image” [10]. In addition to scientifically documenting therapeutic outcomes, HSV has the potential to supplement and replace clinical diagnosis of voice disorders and vocal fold vibratory dysfunction. However, normative data must be established for HSV parameters to increase the therapeutic utility and clinical significance of this powerful imaging technique. One of the initial elements to establish is the effect of HSV recording frame rate on HSV parameters. To our knowledge, no research has examined the effect of HSV recording frame rate on computed quantitative HSV parameters. Nevertheless, as previously said, it is vital to study the behavior and stability of HSV parameters when HSV recording rates change. Consequently, this was the focus of the present endeavor, which aimed to raise awareness of the issue and advocate for the standardization of HSV parameter computation.

The article "Optimal Deep Learning-Based Vocal Fold Disorder Detection and Classification Model on High-Speed Video Endoscopy" was published in 2022. Journal: J Healthc Eng.

This study presents the best deep learning-based vocal fold disorder detection and classification (ODL-VFDDC) method using HSV. The suggested ODL-VFDDC technique employs preprocessing, feature extraction, and feature selection procedures. Furthermore, the obtained characteristics are fed into the deep belief network (DBN) model. Furthermore, the agricultural fertility algorithm (AFA) is employed to optimize the DBN model's hyperparameter tuning, which improves classification results. The farmland fertility algorithm (FFA) is used to gather accurate glottal margins during vocal fold vibrations. The study's goals are to (1) establish a theoretical framework for the proposed model and (2) demonstrate its applicability in practice. (iii) It shows how vocal fold boundaries are represented in HSV data during the linked speech, as well as the tensile strength of demanding colored HSV pictures. As a result, the recommended plan was executed. HSV data was collected from a vocally normal adult using a color high-speed camera. The performance of the ODL-VFDDC model is evaluated using a benchmark dataset, and the findings are examined in a variety of ways.

The remaining section of this paper is structured as follows.  Section 2 contains works that are related.  Section 3 then provides a proposed system description. Then, in Section 4, the detailed performance of the suggested system is shown, and in Section 5, the research work is concluded.

## 2. Related Works

Yousef et al. [11]. The proposed automatic spatial segmentation is a critical step in ushering in a new era of precision laryngeal imaging measurements. This work is required for the automatic extraction and measurement of vocal fold vibratory characteristics. For the whole “Rainbow Passage,” temporal segmentation and motion compensation were able to distinguish the vocalized portions and locate the vibrating vocal folds. The created automated spatial segmentation system successfully captured the vocal fold boundaries across frames for each vocalization, allowing for correct GAW computation at each frame.

The article "Optimal Deep Learning-Based Vocal Fold Disorder Detection and Classification Model on High-Speed Video Endoscopy" was published in 2022. Journal: J Healthc Eng.

Fehling et al. [12] presented a method for autonomously segmenting the time-varying glottal region and vocal fold tissue from laryngeal HSV using the DCNN methodology. The segmentation quality of a higher-performing CNN that considers the temporal environment using LSTM cells.

Using pathological speech recognition and artificial intelligence, Hu et al. [13] discovered novel vocal fold disorders. The method was trained with a CNN model, and the results were compared to those of human experts. This artificial intelligence-based technology might be utilized in medical contexts to detect abnormalities in the vocal folds by simply listening to the person's voice.

Koc et al. [14] proposed an automated approach for segmenting the glottis in images of HSV vocal folds. In HSV photographs, a mask is initially built based on the ROI's overall variation standard. The planar lighting system is then evaluated using consecutive HSV and reflectance images. The masked HSV is used to make an image of the distribution of reflectance in a vertical slice.

Kist and Döllinger [8] performed a complete examination of the U-Net structure in terms of computing load and inference speed by lowering the number of parameters and computations in the approach. At first, the U-Net structure was looked at to see if it could simplify processing, speed up run time, and always keep a higher level of accuracy.

Ali et al. [15] suggested an approach that is based on human hearing and can diagnose and classify a wide range of vocal fold problems. In the current method, important bandwidth phenomena are explored using bandpass filters dispersed over the Bark scale. Kist et al. [16] provided a thorough examination of a method that identifies the glottal midline completely automatically. Then, they created a biophysical system to generate a variety of vocal fold oscillations. Before using these two simulations and the annotated endoscopic images to train DNN at different stages of the study and compare it to the CV method, they also manually annotated the publicly available BAGLS data set.

In contrast to several current spatial segmentation methods, which are more vulnerable to picture noise and intensity uniformity, the suggested ODL-VFDDC approach is noise-resistant. To capture the glottal boundaries in each kymogram, we divided HSV kymograms at various vocal fold cross-sections in individual vocalization using our suggested technique. The kymogram edges were recognized and registered to the HSV frames [17].

## 3. The Proposed Model

In this study, a unique ODL-VFDDC system is developed for categorizing and detecting vocal fold diseases. Preprocessing, feature extraction, feature selection, DBN-based classification, and FFA-based hyperparameter optimization are the steps involved in the proposed ODL-VFDDC approach. The overall process of the ODL-VFDDC technique is depicted in Figure 1.

The article "Optimal Deep Learning-Based Vocal Fold Disorder Detection and Classification Model on High-Speed Video Endoscopy" was published in 2022. Journal: J Healthc Eng.

### 3.1. Preprocessing

The timing of the vibration starts and the offset of vocalized segmentation is automatically recovered from the HSV using temporal segmentation [18]. After noise reduction and motion compensation, the video frame of all vocalizations is used to figure out where the vocal folds are present in the window.

### 3.2. Feature Extraction and Selection

Accurate feature selection is required for the ML technique to be used effectively. In image feature extraction, the texture and intensity of the pixels are the most important factors [19]. The matrix cells (pixels) are composed of three image modules with arithmetic values ranging from 0 to 255. Three features retrieved are a gradient feature and two intensity features. Several combinations of the above-mentioned characteristics are used in the development of the proposed algorithm [20] to find the feature that must be used for executing an accurate depiction of the vocal fold edge. The pixel intensities of the green and red channels are considered two characteristics of the kymogram.

The proper feature selection is a crucial first step in the successful use of the ML approach. The intensities and textures of the pixels play a major role in determining how to extract the characteristics from an image [21]. A 2-D matrix is made up of the pixels in the kymogram's horizontal and vertical directions. The three image components in each matrix (pixel) cell have a numerical value between 0 and 255, which corresponds to the three color channels (i.e., red, green, and blue). The features were calculated using only the intensity values of the red and green channels. The blue channel was excluded from the analysis due to severe noise and a lack of essential data. In this work, two intensity features and a gradient feature were retrieved as three features [22]. The creation of the suggested algorithms used various numbers and combinations of the features to decide which features should be used to provide an appropriate vocal fold edge representation.

Intensity Features: Red and green channel pixel intensities in a kymogram were regarded as two characteristics. Selecting the pixel intensities as a feature was crucial to making it easier to tell the glottal area from the laryngeal tissues in the kymograms since the regions of interest in the kymogram (glottal areas) have lower intensities (darker) than the surrounding regions. Due to the significant degree of noise in the current video data and the occurrence of black pixels outside of the glottis, relying just on intensities as features were insufficient to segment the image.

The article "Optimal Deep Learning-Based Vocal Fold Disorder Detection and Classification Model on High-Speed Video Endoscopy" was published in 2022. Journal: J Healthc Eng.

As the region of interest in kymograms has a lower intensity (darker color) than the surrounding region, it is critical to distinguish the glottal region using pixel intensity [23]. Due to the increasing noise level in the prior video footage and the existence of black pixels, the intensity feature is insufficient to segment the image (except for the glottis). The contrast between the surrounding areas and the intensity of the glottis is used to identify the glottal area borders using an image gradient [24]. The positive and negative gradients in the kymogram are computed with an eight-pixel step size beside *x*-and *y*-axes. As a result, features are extracted using the kymogram image gradient.

### 3.3. DBN-Based Disorder Detection and Classification

DBNs transcend the restrictions of backpropagation by employing unsupervised learning to generate layers of feature detectors that represent the statistical structure of the input data without any prior knowledge of the intended output. High-level feature detectors capture complicated higher-order statistical patterns in input data that may be used to forecast the labels [24]. DBNs based on RBMs are one of the most significant deep learning technologies. RBMs are equivalent to DBN building blocks in that they provide an effective training mechanism. The DBN model is used to identify and categorize vocal folds. The RBM is a blended distribution of visible and hidden units in which the parameters for energy function are set as given below:

(1) $$\begin{array}{c} E\left(v,h,\theta \right)=\underset{j}{\sum }\frac{{\left(v_{j}-C_{i}\right)}^{2}}{2\sigma_{j}^{2}}-\underset{i}{\sum }c_{i}h_{i}-\underset{j,i}{\sum }\frac{v_{j}}{\sigma_{j}}h_{i}W_{ji}, \end{array}$$

where *σ*_*j*_ represents the standard deviation (SD) of Gaussian noise to visible units. As the data are predicted in a usual manner under the speech for spectrograms, it is anticipated that the spectrogram will be converted to a picture to create a comparable dimension. The weighted distribution of the prediction based on real data and the forecast method is determined as shown below:

(2) $$\begin{array}{c} -\frac{\partial \log P\left(v\right)}{\partial W_{ji}}={\langle v_{j}h_{i}\rangle }_{real}-{\langle v_{j}h_{i}\rangle }_{predict}, \end{array}$$

where 〈*v*_*j*_*h*_*i*_〉 represents the distribution's expected value, as stated by the subscript that follows. The stochastic ascent from the log probability of learned data is proven using a simple rate of learning concept as follows:

(3) $$\begin{array}{c} \Delta W_{ji}=\alpha \left({\langle v_{j}h_{i}\rangle }_{real}-{\langle v_{j}h_{i}\rangle }_{predict}\right). \end{array}$$

The pace of learning is denoted by the symbol. The purpose of applying the DBN's learning rate for locating momentum from upgrading weight and bias. MLP uses DBN's infrastructure, which is divided into many tiers. The DBN approach uses feature extraction in signal representation to train the infrastructure system, which was the basic conceptual design [25]. One of the main goals of trained DBN is to train a stack of RBMs, whereas the model of parameters *θ* learned by probability determines both *P*(*v|*h; *θ*) and the previous distribution on hidden vector (*h|θ*), thus the probability of visible vector (*v*)î expressed as:

(4) $$\begin{array}{c} P\left(v\right)=\underset{h}{\sum }P\left(h|\theta \right)P\left(v|h;\theta \right). \end{array}$$

After learning *θ* the previous probability of *P*(*v|h*; *θ*)*is* reserved but *P*(*h|θ*) is exchanged by maximizing the frame level of cross entropy using the class label's forecast probability distribution. This replacement enhances the likelihood of training in composite models by reducing different constraints [26]. The DBN framework is shown in Figure 2.

The article "Optimal Deep Learning-Based Vocal Fold Disorder Detection and Classification Model on High-Speed Video Endoscopy" was published in 2022. Journal: J Healthc Eng.

DBN training is often divided into two stages: greedy layer-wise pretraining and practice fine-tuning. Unsupervised training and farmland fertility method (FFM) are used to train the model parameters layer by layer in layer-wise pretraining [27]. The training begins with the lower-level RBM that receives the DBN inputs and progresses up the hierarchy until it reaches the top-level RBM that stores the DBN outputs. As a consequence, the preceding layer's learned features or output is used as input for the subsequent RBM layer. Following the training of RBM, the network may be fine-tuned in a supervised manner using the backpropagation approach as the last step.

Data were collected while a vocally healthy person recited the “Rainbow Passage” using a specially constructed HSV system [28]. The glottal area in the HSV data was segmented using a deep belief network (DBN). The glottis region was automatically tagged during vocal fold vibrations using a recently developed hybrid approach by the authors as an automated labeling tool to train the network on a series of HSV frames. The network was then evaluated on various phonatory events on the HSV sequence using multiple metrics, including intersection over union (IoU) and boundary F1 (BF) score, against manually segmented frames. Therefore, DBN structures are recognized as RBMs, which generate the unit variable from a directional network and fix a quick-assessed prediction with a collection of detection weights. For DBN processing, it is defined as a peak in a waveform [29–32]. It is not as easy as utilizing the FFT to digitally alter the data to establish a peak of raw waveform signals. The staging approach searching for peaks is as follows:

- Initializing length of window signals *X*.
- Divided the signal frame into 3 sections right, left, and center.
- Implementing any function (min, median, max, mean, and so on.)
- Verify the maximal center value in the peak. Choose maximal value *f*(*c*) extremely closer to the window, define the peak then mark it and endure. Else, go to the next step.
- Alteration of input data by one instance and repeat the procedure.
- When all data are being processed, the peaks are identified.

The article "Optimal Deep Learning-Based Vocal Fold Disorder Detection and Classification Model on High-Speed Video Endoscopy" was published in 2022. Journal: J Healthc Eng.

After that, determine the peaks of the waveform and run the DBN proposal with input and output dimensions set, and set up the windowing frame vector for fixed value modification of the DBN's minimal layer's visible unit, which means generating a probability distribution on the prediction label [33–35]. The hammer distance technique is used to anticipate the likelihood of future possibilities.

### 3.4. Hyperparameter Tuning Using FFA

The FFA is used to optimize the setting of the DBN model's hyperparameters. The FFA method solves the optimum problem by simulating farmers' performance while applying different fertilizers on farms with varying soil quality. The fertilizing approach to the land is the same throughout this technique, and the soil quality is equal to the fitness worth of humans. For land with poor soil quality, an ideal fertilization plan is chosen, but the fertilization design for other land is chosen at random [32]. The continuous advancement of fertilization processes successfully enhances agricultural soil quality.

Algorithm 1 demonstrates the pseudocode of FFA. The key stages are described in detail below. It can be assumed that the number of individuals is *N*, and all individuals *X*_*i*_ are demonstrated as *X*_*i*_=[*X*_*i*1_, *X*_*i*2_, *X*_*i*3_,…, *X*_*iD*_](*i*=1,2,…, *N*), where *D* refers to the dimensional of optimizing problem, *X*_*ij*_(*j*=1,2,…, *D*) refers the value of *i*^*th*^ individuals from the *j*^*th*^ dimension and *N* refers the individuals arbitrarily created using:

(5) $$\begin{array}{c} X_{ij}=L_{j}+rand\times \left(U_{j}-L_{j}\right), \end{array}$$

where *U*_*j*_ and *L*_*j*_ are the upper and lower limits of the optimized problems searching ranges, respectively. A rand is an arbitrary number between zero and one. The following is a method of partitioning the farming region. The people were first numbered. Following that, *n* number of consecutive people are segregated into one zone depending on the primary person; however, it might be equally separated into *k* sections [36]. The value of *k* is an integer more than 2 but less than 4; when no specific conditions are specified, if *k* = 4, this approach achieves an excellent result.

The article "Optimal Deep Learning-Based Vocal Fold Disorder Detection and Classification Model on High-Speed Video Endoscopy" was published in 2022. Journal: J Healthc Eng.

The person made from people from all around the world is shown by,

(6) $$\begin{array}{c} s_{a}=\left\{x_{\left(a-1\right)\times n+1},x_{\left(a-1\right)\times n+2},\ldots ,x_{\left(a-1\right)\times n+n}\right\},\left(a=1,2,\ldots ,k\right), \end{array}$$

where *a* implies the sub-region number, that is, *a* ∈ [1, *k*], and *a* ∈ *N*^+^; *n*=*N*/*k*; *S*_*a*_ implies the group of individuals comprised in the region *a*. In order to minimize problems, the area with worse average soil *S*_worst_ signifies the region with maximum average fitness value of individual and vice-versa. The particular computation is demonstrated as follows:

(7) $$\begin{array}{c} S_{worst}=arg\;\max\left\{Fit_{a}=\frac{\overset{n}{\underset{i=1}{\sum }}f\left(S_{a}\left(i\right)\right)}{n}\right\}, \end{array}$$

whereas fit (*S*_*a*_(*i*)) refers to the fitness value of *i*^*th*^ individual from region *a*.

The memory comprises local and global memory. A primary *M*_*L*_ individual with higher soil quality from all the regions is saved from the local memory, but the primary *M*_*G*_ individuals with higher soil quality from the total area are saved from the global memory. *M*_*L*_ and *M*_*G*_ are defined using the subsequent formulas:

(8) $$\begin{array}{c} M_{L}=round\left(t\times n\right), \end{array}$$

(9) $$\begin{array}{c} M_{G}=round\left(t\times N\right), \end{array}$$

where *t* refers to the arbitrary number between 0.1 and 1, and round represents the rounding outcome.

Individuals from low-quality soil sub-region and individuals from other subregions are employed to optimize the soil [37, 38]. Here is an example of a well-optimized technique. As depicted by an individual, it employs one of the most successful fertilization procedures for spawning new individuals in order to enhance the soil quality of the poorest region as much as possible.

(10) $$\begin{array}{c} X_{inew}=h_{1}\times \left(X_{i}-X_{MGlobal}\right)+X_{i},\left(i=1,2,\ldots ,n\right), \end{array}$$

where *X*_*M*Global_ signifies the arbitrarily chosen individual in the global memory, and *h*_1_ is computed as follows:

(11) $$\begin{array}{c} h_{1}=\alpha \times rand_{1}, \end{array}$$

where *α* represents the constants, that is, *α* ∈ [0,1], and rand_1_ indicates the arbitrary number between −1 and 1.

Novel people are developed using the following method to create individuals from places other than the region with the worst soil quality:

(12) $$\begin{array}{c} X_{inew}=h_{2}\times \left(X_{i}-X_{u}\right)+X_{i},\left(i=1,2,\ldots ,n\right), \end{array}$$

where *X*_*u*_ indicates the individual chosen arbitrarily in every individual and *h*_2_ is computed as follows:

(13) $$\begin{array}{c} h_{2}=\beta \times rand, \end{array}$$

where *β* represents the constant, that is, *β* ∈ [0,1] and *rand* denotes the arbitrary number between *zero* and one.

The article "Optimal Deep Learning-Based Vocal Fold Disorder Detection and Classification Model on High-Speed Video Endoscopy" was published in 2022. Journal: J Healthc Eng.

All the individuals *X*_*i*_ are fused with an optimum individual from global or local memory by utilizing

(14) $$\begin{array}{c} X_{inew}=\left\{\begin{array}{cc} X_{i}+\omega_{1}^{d}\times \left(X_{i}-G\left(B\right)\right)\text{,} & Q>rand\text{,}\\ X_{i}+rand\times \left(X_{i}-L\left(B\right)\right), & else\text{,} \end{array}\right. \end{array}$$

where *G*(*B*) and *L*(*B*) signify the optimum individual from the global and local memory of all the regions, respectively; *Q* represents the constant, for instance, *Q* ∈ [0,1], and their value is usually 0.7 if no specific instruction is provided; rand signifies the arbitrary number between zero and one; and *ω*_1_^*d*^ is *ω*1 at *d*^th^ iteration and reduces with iteration procedure according to the subsequent formula:

(15) $$\begin{array}{c} \omega_{1}^{d+1}=\omega_{1}^{d}\times rand, \end{array}$$

where *ω*_1_^1^ is *ω*_1_ implies the custom integer, an initial iteration, and usually equivalent to 1 for obtaining better results.

## 4. Results and Discussion

The performance validation of the ODL-VFDDC model is examined in this section. The results are examined using a variety of test photos gathered from various sources. Python 3.6.5 is used to simulate the proposed ODL-VFDDC model.  Figure 3 shows some examples of pictures.

In Table 1 and Figure 4 show the ODL-VFDDC model's outcome analysis for various parameters and runs. Initial frequency, jitter, shimmer, and HNR are four separate factors that are examined in the results. The ODL-VFDDC model produced effective vocal fold disorder classification results in every run, according to the experimental results and sample figure shown in Figures 3(a) and 3(b).

For example, under run 1 and beginning frequency, for example, the ODL-VFDDC model has an accuracy, sensitivity, and specificity of 58.49%, 57.30%, and 61.86%, respectively. Under run 1 and jitter, the ODL-VFDDC model exhibits sensitivity, accuracy, and specificity of 97.20%, 77.23%, and 16.71%, respectively. Under running 1 and HNR, the ODL-VFDDC model achieved sensitivity, accuracy, and specificity of 71.46%, 64.66%, and 55.02%, respectively. Furthermore, under run 3 and beginning frequency, the ODL-VFDDC technique generated accuracy, sensitivity, and specificity of 58.16%, 58.11%, and 60.68%, respectively. Under run 3 and jitter, the ODL-VFDDC technique similarly exhibits accuracy, sensitivity, and specificity of 77.69%, 96.82%, and 18.37%, respectively. The ODL-VFDDC algorithm has a sensitivity, accuracy, and specificity of 70.20%, 65.95%, and 65.95%, respectively as shown in Figure 5.

The article "Optimal Deep Learning-Based Vocal Fold Disorder Detection and Classification Model on High-Speed Video Endoscopy" was published in 2022. Journal: J Healthc Eng.

In terms of accuracy, recall, and *F* measure, Figure 6 compares the ODL-VFDDC methodology to previous methodologies. According to the data, the DT system performed badly, with accuracy, recall, and F measure values of 92.19%, 93.02%, and 93.12%, respectively.

Furthermore, the Conv-NN model performs somewhat better, with accuracy, recall, and *F* measures of 95.90%, 96.06%, and 97.38%, respectively. The KNN and FCBD models then provided findings that are comparable. After that, the FCB strategy got a near-optimal recall, precision, and *F* measures of 98.46%, 96.07%, and 97.64%, while the ODL-VFDDC strategy got good results with measures of 97.53%, 99.07%, and 98.89% for precision, recall, and *F* measures, respectively.

Table 2 and Figure 7 depict a brief comparison of the ODL-VFDDC model to other techniques. According to the data, the decision tree model performed worse, with an accuracy of 92.04 percent. Furthermore, the Conv-NN model has somewhat increased performance, with a 95.12 percent accuracy. Furthermore, the KNN and FCBD techniques were somewhat more accurate, with 97.96% and 97.17% accuracy, respectively. Finally, whilst the FCB approach produced a near-optimal accuracy of 98.29%, the supplied ODL-VFDDC system produced an effective outcome with an accuracy of 98.95%.

Finally, Table 3 and Figure 8 show a detailed execution time study of the ODL-VFDDC model. According to the data, the Conv-NN model delivered inadequate results with a minimum execution time of 280 ms.

The DT and KNN models, on the other hand, yielded marginally faster execution durations of 55 and 52 milliseconds, respectively. Furthermore, the FCB and FCBD models dramatically reduced execution times to 47 and 43 milliseconds, respectively. With a 25 ms execution time, the ODL-VFDDC model outperformed the other techniques. From the facts and tables above, it is clear that the ODL-VFDDC model did better than the others.

The DT and KNN models then produced reaction times of 67 and 42 milliseconds, respectively. Furthermore, the FCB and FCBD models considerably reduced execution times to 39 and 35 milliseconds, respectively. With a 20 ms execution time, the ODL-VFDDC model outperformed the other approaches as shown in Table 4. By looking at the numbers and tables above, it is clear that the ODL-VFDDC model did better than the others.

The article "Optimal Deep Learning-Based Vocal Fold Disorder Detection and Classification Model on High-Speed Video Endoscopy" was published in 2022. Journal: J Healthc Eng.

Figure 9 depicts an MSE analysis of the ODL-VFDDC model in contrast to previous techniques. According to the data, the Conv-NN model performed worse, with an MSE of 66.04 percent. Furthermore, with an MSE analysis of 35.12%, the FCDB model's performance has been somewhat enhanced. Furthermore, the decision tree, KNN, and FCB methods were slightly closer, with MSE analyses of 57.96%, 42.81%, and 39.17%, respectively. In the end, the suggested model ODL-VFDDC system worked well, with an MSE of 19.92% or less.

## 5. Conclusion

In this work, a novel ODL-VFDDC approach was created for identifying and categorizing vocal fold dysfunction. The suggested ODL-VFDDC technique includes preprocessing, feature extraction, feature selection, DBN-based classification, and FFA-based hyperparameter optimization. The performance of the ODL-VFDDC model is validated using a benchmark dataset, and the results are evaluated in a variety of ways. In terms of vocal fold disorder classification, the results demonstrated that the ODL-VFDDC technique beat the other current methodologies. When applied to tough HSV data taken with a color camera, the suggested strategy produced positive results, paving the way for increased accuracy and performance when applying the ODL-VFDDC method on less difficult photos (monochromatic images). Given the limits of endoscopic analysis of linked speech, the ODL-VFDDC technique might be a useful tool for automating the results and performance of vocal fold dynamics. As a result, the ODL-VFDDC technique has improved vocal fold disease classification. The ODL-VFDDC technique achieved an accuracy of 98.95%, F score of 98.89%, recall of 99.07%, and AP rate of 99.07%. A hybrid technique of RBMs, DBNs, and LSTMs will be used as a preprocessing approach in the future to see if it significantly improves the DBN's performance.

## Figures and Tables

**Figure 1:** The overall process of the ODL-VFDDC technique.

**Figure 2:** The framework of DBN.

**Figure 3:** (a). Sample images (normal) and (b). sample images (abnormal).

**Figure 4:** Result analysis of the ODL-VFDDC technique under distinct parameters and runs.

**Figure 5:** AP and RP rate analysis of the ODL-VFDDC technique with recent algorithms.

**Figure 6:** Comparative analysis of ODL-VFDDC technique with recent algorithms.

**Figure 7:** Accuracy analysis of the ODL-VFDDC technique with recent algorithms.

**Figure 8:** Execution time analysis of the ODL-VFDDC technique with recent approaches.

**Figure 9:** MSE analysis of the ODL-VFDDC technique with recent approaches.

**Algorithm 1:** : Pseudocode of FFA.

**Table 1:** Result analysis of ODL-VFDDC technique under distinct parameters and runs.

Parameters	Accuracy	Sensitivity	Specificity
*Run-1*			
Initial frequency (*F*_o_)	58.49	57.30	61.86
Jitter (%)	77.23	97.20	16.71
Shimmer (%)	79.00	93.61	34.15
HNR (dB)	64.66	71.46	55.02
Average	**69.85**	**79.89**	**41.94**

*Run-2*			
Initial frequency (*F*_o_)	60.21	59.49	62.01
Jitter (%)	77.97	97.62	15.79
Shimmer (%)	76.48	95.67	34.67
HNR (dB)	68.03	71.30	57.18
Average	**70.67**	**81.02**	**42.41**

*Run-3*			
Initial frequency (*F*_o_)	58.16	58.11	60.68
Jitter (%)	77.69	96.82	18.37
Shimmer (%)	78.56	95.45	34.08
HNR (dB)	65.95	70.20	55.40
Average	**70.09**	**80.15**	**42.13**

*Run-4*			
Initial frequency (*F*_o_)	58.42	57.92	61.09
Jitter (%)	78.47	99.09	17.18
Shimmer (%)	76.89	93.52	35.10
HNR (dB)	64.65	68.84	56.84
Average	**69.61**	**79.84**	**42.55**

*Run-5*			
Initial frequency (*F*_o_)	59.21	57.71	62.71
Jitter (%)	77.79	98.05	17.87
Shimmer (%)	77.75	94.03	34.37
HNR (dB)	66.10	70.35	56.56
Average	**70.21**	**80.04**	**42.88**

The article "Optimal Deep Learning-Based Vocal Fold Disorder Detection and Classification Model on High-Speed Video Endoscopy" was published in 2022. Journal: J Healthc Eng.

**Table 2:** Comparative analysis of the ODL-VFDDC technique with recent approaches.

Methods	AP rate	EP rate	Precision	Recall	*F* measure	Accuracy
Decision tree model	93.02	6.98	92.19	93.02	93.12	92.04
Conv-NN model	96.06	3.94	95.90	96.06	97.38	95.12
KNN model	97.20	2.80	95.95	97.20	98.34	97.96
FCB model	98.45	1.56	96.07	98.45	97.64	98.29
FCBD model	97.10	2.90	94.46	97.10	97.93	97.17
ODL-VFDDC	99.07	0.93	97.53	99.07	98.89	98.95

**Table 3:** Execution time analysis of the ODL-VFDDC technique with current technologies.

Methods	Execution time (ms)
Decision tree model	55
Conv-NN model	280
KNN model	52
FCB model	47
FCBD model	43
ODL-VFDDC	25

**Table 4:** Response time analysis of the ODL-VFDDC technique with current technologies.

Methods	Response time (ms)
Decision tree model	67
Conv-NN model	153
KNN model	42
FCB model	39
FCBD model	35
ODL-VFDDC	20

## Data Availability

The manuscript contains all data.
